The article "An In Vivo Study of Lactobacillus rhamnosus (PTCC 1637) as a New Therapeutic Candidate in Esophageal Cancer" was published in 2022. Journal: Biomed Res Int.

# An In Vivo Study of *Lactobacillus rhamnosus* (PTCC 1637) as a New Therapeutic Candidate in Esophageal Cancer

**DOI:** 10.1155/2022/7607470

**Published:** 2022-06-24

**Authors:** Malihe-sadat Hashemi-Khah, Nazila Arbab-Soleimani, Mohammad-Mahdi Forghanifard, Omid Gholami, Saba Taheri, Sakineh Amoueian

**Affiliations:** ^1^Department of Microbiology, Damghan Branch, Islamic Azad University, Damghan, Iran; ^2^Department of Biology, Damghan Branch, Islamic Azad University, Damghan, Iran; ^3^Cellular and Molecular Research Center, Sabzevar University of Medical Sciences, Sabzevar, Iran; ^4^Department of Biology, Islamshahr Branch, Islamic Azad University, Islamshahr, Iran; ^5^Pathology Department, Emam Reza Hospital, Mashhad University of Medical Sciences, Mashhad, Iran

## Abstract

**Objective:**

This study is aimed at investigating the effect of probiotic *Lactobacillus rhamnosus* on esophageal cancer *in vivo* and *in vitro*.

**Methods and Results:**

In this study, the cytotoxicity effects of *L. rhamnosus* supernatant and whole-cell culture on a cancer cell line (Kyse30) compared to 5fu were evaluated by the MTT assay. The real-time PCR method was used to analyse the *L. rhamnosus* supernatant effect on the expression of Wnt signaling pathway genes. An *in vivo* investigation in nude mice was done to assess the anti-tumor activity of *L. rhamnosus* supernatant and whole-cell culture. Both supernatant and whole-cell culture of *L. rhamnosus* reduced cell survival (Kyse30) *P* < 0.001. The supernatant of this bacterium significantly reduced the expression of Wnt signaling pathway genes. Administration of supernatant and whole-cell culture of *L. rhamnosus* expressively reduced tumor growth compared to the control group. The effects of this bacterium on tumor necrosis were quite evident, pathologically *P* < 0.01.

**Conclusion:**

This study is the first report that assessed the potential impact of *L. rhamnosus*, especially its supernatant on esophageal cancer and Wnt signaling pathway genes. Therefore, this bacterium can be a harmless candidate for esophageal cancer therapy.

## 1. Introduction

Esophageal cancer is a malignancy in the esophagus tissue spread in developing countries. This cancer is divided into two types: (1) squamous cell carcinoma, which appears in the middle or top of the esophagus and (2) adenocarcinoma, seen in the glandular cells of the esophagus [1]. Symptoms such as chronic cough, indigestion, vomiting, fatigue, and heartburn appear during cancer progression [2, 3]. It is believed that mutations in the deoxyribonucleic acid (DNA) signal the cells related to the esophagus to multiply abnormally [4, 5].

Generally speaking, signal transduction pathways in the initiation and progression of cancer are essential. Thus, targeting signal molecules can be helpful for cancer therapy [6]. The Wnt pathway is one of the most critical signaling pathways activated by mutation in many cancers [7–9]. This signaling pathway plays essential roles in different cellular processes, including stem cell maintenance, differentiation, migration, apoptosis, and proliferation. Abnormal activation of the Wnt cascade leads to carcinogenesis [10, 11]. The Wnt cascade consists of canonical and non-canonical pathways, of which the former is believed to be involved in self-regeneration. In the absence of Wnt signals, the cytoplasmic catenin beta-1 (*β-catenin*) is associated with a complex including auxin, *glycogen synthase kinase 3* (*GSK-3*), and *adenomatous polyposis coli* (*APC*) (the *APC* protein acts as the primary regulator of *β-catenin* function). Upon binding to this complex, *β*-catenin is phosphorylated, thus being labeled for degradation in the proteasome. In the presence of Wnt signals, the Wnt proteins bind to (frizzled) *frizzled receptors* (*FZDs*) and *low-density lipoprotein receptor-related protein* (*LRP*) receptors, leading to the stabilization of *β-catenin*, its transfer to the nucleus, and the activation of target genes. *β-catenin* forms a complex with T-cell factor (*TCF*)*/lymphoid enhancer factor* (*LEF*) transcription factors and cofactors such as histone acetyltransferase p300 (p300), CBP, BCL9, and pygopus, to transcribe Wnt signaling target genes such as *Cyclin D1*, *C-Myc*, and *survivin* [9, 12–15].

Lactic acid bacteria, especially *lactobacilli* with probiotic potential, are known as promising tools for cancer therapy. Cancer-preventing strategies of these beneficial bacteria such as binding to carcinogens and degrading them, stimulating anti-cancer enzymes, and preventing the conversion of procarcinogens to carcinogens, production of beneficial compounds that act as signaling molecules affecting the immune system, cell death, and proliferation, and interference with cell signaling pathways are reported [16–19]. Recently, the significant effects of whole-cell components and supernatants of probiotic *lactobacilli* in the prevention, suppression, and treatment of many cancers (lung, colon, breast, colorectal, stomach, etc.) have been considered [20].

This study was designed to investigate the effect of probiotic *Lactobacillus rhamnosus* (*L. rhamnosus*) on the expression of the Wnt signaling pathway genes and esophageal cancer as a harmless therapeutic candidate.

## 2. Material and Methods

### 2.1. Ethical Statement

This study was approved by the Islamic Azad University, Damghan Branch, Ethical Committee (Approval ID: IR.IAU.DAMGHAN.REC.1398.003) (https://ethics.research.ac.ir/EthicsProposalView.php?id=60331).

### 2.2. Bacterial Strain

A standard strain of *L. rhamnosus* (PTCC 1637) was acquired from Persian Type Culture Collection and cultivated in Man-Rogosa-Sharpe (Merck, Germany, Cat#: 110661) broth for 24-48 hours at 37°C in anaerobic conditions.

### 2.3. Preparation of Cell-Free Supernatant

To prepare cell-free supernatant (CFS), probiotic *Lactobacillus* was cultivated in an MRS broth medium for 24 h at 37°C. CFS was obtained by centrifuging the culture (4°C, 10000 rpm, 10 min), followed by filtration of the supernatant through a 0.2 *μ*m pore size filter [21, 22].

### 2.4. Cell Line

The human esophageal squamous cell carcinoma (ESCC) cell line KYSE-30 was acquired from the Pasteur Institue and cultured in RPMI-1640 medium (BioIdea, Cat#: BI-1006-05) with stable glutamine, supplemented with 10% (*v*/*v*) fetal bovine serum (FBS) (BioIdea, Cat#: BI-1201), 100 U/mL penicillin, and 100 *μ*g/mL strept. The cell line was grown at 37°C with 5% CO2 in a humidified environment of 95% [23].

### 2.5. *In Vitro* Cytotoxic Assay

The cytotoxic effects of *L. rhamnosus* (whole-cell culture and supernatant) and 5-FU on the KYSE-30 cell line were determined by 3-(4,5-dimethylthiazol-2-yl)-2,5-diphenyl tetrazolium bromide (MTT) assay. Briefly, KYSE-30 cells were seeded at a density of 5000 cells/well in a 96-microtiter plate and incubated for 24 hours. The cells were treated with different concentrations of whole-cell culture and CFS of *L. rhamnosus* (2.5-320) mg/ml and 5-FU (0.312-320) mg/ml for 24, 48, and 72 hours. Then, 20 *μ*l MTT (DNAbiotech, Cat#: DMA500) solution (final concentration of 5 mg ml^−1^) was added to the wells and incubated for 4 hours at 37°C. Finally, 100 *μ*l dimethyl sulfoxide (DMSO) was added, and the optical density of each well was read at 570 nm using ELISA plate reader (STAT Fax-USA, Model: Z100). To assess the cell viability, the absorption of drug-treated cells was divided by the absorption of control (non-drug) cells and multiplied by 100 [24–27]. Analyses were done using GraphPad prism version 5 software.

### 2.6. Ribonucleic Acid (RNA) Extraction and Comparative Real-Time PCR

TRIzol reagent (DNAbiotech, Cat#: DB9683) was used to extract RNA from treated and control KYSE-30 cells in accordance with the manufacturer's instructions. Cells were rinsed in phosphate-buffered saline (PBS), then incubated at room temperature for 15 minutes with TRIzol reagent (1000 *μ*l). Chloroform (200 *μ*l) was added to the samples, mixed gently, and incubated for 15 minutes at room temperature. After incubation, the samples were centrifuged for 15 minutes at 4°C at 13,000 rpm. After centrifuging at 13,000 rpm for 10 minutes, RNA was precipitated from the aqueous phase by adding isopropyl alcohol to a new tube containing the supernatant aqueous phase. Gel electrophoresis and nanodrop (Nano100; Bio Intellectica, Canada) were employed to assess the purity and amount of RNAs, respectively. To make cDNA, a PrimeScript First Strand cDNA Synthesis Kit (Yekta Tajhiz Azma, Cat#: YT4500) was utilized. The SYBR Green technique was used to do comparative relative real-time PCR in triplicates using the Stratagene Mx3000P. Oligo7 program created the primer sets that were utilized (Table 1). The real-time PCR temperature profile was as follows: 95°C (10 min), 39 cycles at 95°C (15 s), 60°C (20 s), and 72°C (20 s). The 2^−ΔΔCt^ technique was used to assess fold changes in gene expression using the actin housekeeping gene as a normalizer [28, 29].

### 2.7. Animal Experimentation

All tests were carried out according to the protocol authorized by the Ethical Committee of Islamic Azad University's Damghan Branch. Twenty-four nude mice (15 ± 5 g, 5 to 6 weeks of age) were purchased from the Pasteur Institute of Tehran and divided into four (*n* = 6). Standard maintenance conditions were 18-22°C, 20-25% humidity, and 12 hours of light/dark cycles with free access to water and food before and during the experiments [30].

#### 2.7.1. Tumors and Prescribing Drugs

To cause a tumor tissue, diluted KYSE-30 cells (5 × 10^6^ cells) were injected into the mice on the flank (right side). As follows, the animals were separated into four groups (*n* = 6). The control group (no treatment) and three treatment groups were each given a single dosage of 2 and 3 mg/kg of 5 FU, whole-cell, and CFS of *L. rhamnosus* intraperitoneally for 15 days. After one week, the tumor volume was measured (once every two days) in three directions of length, width, and height, and the assessment of tumor volume was applied through the formula [31]:

(1) $$\begin{array}{c} \left(\text{Length}\times \text{Width}\times \text{Height}\right)\times 0.52 \end{array}$$

For data analysis, one-way ANOVA was followed. (All analyses were done using GraphPad Prism Version 5 for Windows).

#### 2.7.2. Histopathological Study

After scarifying mice of each group on days 5, 10, and 15, the tumor sample was removed and placed in 10% formalin for pathological studies. 4 mm thick sections were cut and put on glass slides. According to the usual procedure in pathology laboratories, a microscopic slide was prepared and stained with hematoxylin and eosin stain (H&E stain) staining, and the necrosis inside the tumor tissue was evaluated. The enumeration of desired factors, including tumor cells and necrotic cells in 9 fields of view, was randomly studied by light microscope [26, 30].

### 2.8. Statistical Analysis

Gene expression results were one-way ANOVA was followed by Tukey's posttest. Results were expressed as mean ± SEM. Statistical significance was defined as *P* values < 0.05 (^∗^*P* < 0.05; ^∗∗^*P* < 0.01; ^∗∗∗^*P* < 0.001). All analyses were performed using GraphPad Prism Version 5 for Windows (GraphPad Software, San Diego, CA).

## 3. Results

### 3.1. MTT Cytotoxic Assay

Cell viability of KYSE-30 cells was measured with the MTT assay. The cells were treated with different concentrations of 5fu, *L. rhamnosus* supernatant, and whole-cell culture of *L. rhamnosus* (0.312–320 mg/ml) for 24, 48, and 72 h (Figure 1). The highest inhibitory effects were observed at the concentrations of 5, 10, 20, and 40… for 5fu (Figure 1(a)), concentrations of 120, 160, 240, and 320 (mg/ml) for *L. rhamnosus* supernatant (Figure 1(b)), and whole-cell culture of *L. rhamnosus* (Figure 1(c)). The exposures of 48 and 72 h were more effective on viability reduction. IC50s (drug concentration that causes 50% mortality) for 48 and 72 h treatment were calculated; they were 2.3 and 1.8 (mg/ml) for 5fu (Figure 1(a)), 119.6 and 116.2 (mg/ml) for *L*. *rhamnosus* supernatant (Figure 1(b)), and 109.4 and 83.5 (mg/ml) for *L*. *rhamnosus* whole-cell culture (Figure 1(c)). The results are expressed as mean ± SEM (*n* = 3). ^∗∗∗∗^*P* < 0.0001.

### 3.2. Wnt Signaling Pathway Gene Expression Analysis

*L. rhamnosus* supernatant significantly reduced expression of the selected genes (*β-catenin*, *GSK*, *FZD*, *TCF-7*, *Cyclin-D*, *APC*, *LRP6*, *LRP5*, *LEF*, *Myc*, and *Wnt1* genes), compared with the 5fu (Figure 2). The *P* value of 5fu and *L. rhamnosus* supernatant was equal to 0.0391 (*P* < 0.1) and 0.0001 (*P* < 0.0001), respectively, in most of the Wnt signaling pathway genes.

### 3.3. Tumor Growth and Final Volume

Results showed that tumor growth was lower in the groups receiving 5fu and *L. rhamnosus* (CFS and whole-cell culture) than in the control group. Tumor growth had a decreasing slope in the treatment receiving groups of *L. rhamnosus* (CFS and whole-cell culture) compared to the control group (*P* value < 0.001) (Figure 3). The statistical analysis was performed including all groups; ^∗∗∗^*P* < 0.001 versus the control group, versus the individual treatment group.

### 3.4. Histopathological Results

Due to the reduction of tumor growth, histopathological results in all three times of tissue sampling showed the amount of necrosis inside the tumor owed to amplified antitumor responses in the 5fu, *L. rhamnosus* (CFS), and whole-cell culture-receiving groups as opposed to the control group. Examination of pathological data shows the reduction of tumor forms and the increase of necrosis (Figure 4).

### 3.5. Tissue Necrosis

Necrosis is a sign of cell death in which the nucleus is completely compressed, the cytoplasm of the cell is completely degraded, and the nucleus is seen as a round thing with a smooth and gathered margin. This condition in cancer cells indicates treatment and the death of cancer cells. Our data showed that prescribing 5fu and *L. rhamnosus* whole-cell culture and its supernatant increases cancer cell necrosis by enhancing antitumor responses in drug-treated mice compared to the control group. There was a significant difference between the control group and the other study groups. Values are expressed as mean ± SEM. ^∗∗^*P* < 0.01 (Figure 5).

## 4. Discussion

Esophageal cancer is a severe malignancy concerning mortality and prognosis. It is a growing health concern and is expected to increase over the next 10 years [32, 33]. The main feature of cancer cells is uncontrolled cell proliferation [34]. Different signaling pathways are active in different periods of human life and naturally cause human evolution and growth. The impairment in the expression and function of factors related to these pathways leads to disorders and diseases such as cancer [7, 8]. Nowadays, cellular messaging pathways have played a significant role in cancer treatment [6]. The Wnt signaling pathway is abnormally activated in various cancers, which is vital in their carcinogenesis progress [35]. Over the past three decades, significant progress has been made in understanding the molecular components and regulation of the Wnt pathway. Considering the complex role of Wnt signaling in cancer, there remain several challenges in setting treatment strategies for the Wnt pathway in certain malignant conditions. Nevertheless, pathway targeting factors indicate a reasonable goal of anti-cancer research [10, 11, 36, 37]. Moreover, according to Moghbeli et al., cellular messaging pathways have played a significant role in preventing tumorigenesis and metastasis [6]. Many cancer therapies, such as chemotherapy, are limited because of their toxic effects on the body's cells and normal tissues. However, probiotics and their derivatives destroy tumor cells without damaging normal cells or having other side effects [38, 39].

*Lactobacilli* are the most common microorganisms used as probiotics, and the anti-tumor properties of these bacteria are proven. They inhibit cancer cell proliferation through their cytoplasmic extracts, heat-killed cells, and cell wall peptidoglycans [40–43]. In addition, their modulatory effects on the cancer-related signaling pathways, apoptosis, metastasis, and cell cycle control were shown [44].

We investigated the effect of cell-free supernatant and whole-cell culture of *L. rhamnosus* against Kyse-30 cancer cells in esophageal cancer and the expression of genes involved in the Wnt pathway. Based on MTT test results, the supernatant and the whole-cell culture of *L. rhamnosus* have anticancer properties, significantly killing cancer cells (*P* < 0.05). The exact reported data by Kim et al. shows that lactic acid bacteria's cytoplasmic extracts and peptidoglycan have anti-proliferative activity against cancer cells in *in vivo* and *in vitro* conditions [45]. Probiotics boost the immune system's anti-inflammatory activities, and their long-term use significantly contributes to the suppression and proliferation of cancers [46]. Research in animal models and cancer cells indicated the anti-tumor effects of probiotics *Lactobacillus casei* and its peptidoglycans [46, 47]. *L. casei* and *L. rhamnosus GG* inhibited RT112 and MGH bladder cancer cells [48]. Different concentrations of heat-killed and supernatant of *Lactobacillus plantarum* A7 and *L. rhamnosus* GG showed reduced bioavailability and cell proliferation in normal and cancer cell lines. Bioactivity at the highest concentrations on HT-29 cells by *Lactobacillus plantarum* and *L. rhamnosus GG* was reported to be about 50% and 62.7%, respectively [49]. Moreover, the cytoplasmic extracts of *L. casei* and *Bifidobacterium* directly affected the growth of cancer cell lines. Thus, at a 50 *μ*l/ml concentration, they inhibited the growth of approximately 50% of cancer cells [50]. *L. rhamnosus* could orally reduce the course of tumor growth and tumor growth rate compared to the control group [30]. This bacterium can inhibit tumor growth rate by affecting genes involved in signal transduction pathways. In our data, *L. rhamnosus* supernatant significantly reduces the expression of different genes, *GSK*, *FZD*, *TCF-7*, *Cyclin-D*, *APC*, *LRP6*, *LRP5*, *Myc*, *Wnt1*, and *LEF*, except for *β-catenin* through Wnt signaling pathways compared to 5fu drug (*P* < 0.05). Other probiotic strains have an inhibitory effect on various biomarkers, and these microorganisms reduce the expression of many molecular markers. *Lactobacilli* prevent tumor growth by targeting the Wnt/*β*-catenin pathway [51, 52]. Yan and Polk showed that solution compounds secreted by *L. casei* and *L. rhamnosus* cause apoptosis in monocytic leukemia cells, so probiotic *Lactobacilli* can be considered a safe agent to battle cancer [53].

From this perspective, lactic acid bacteria with probiotic potentials, such as *L. rhamnosus*, can be a proper candidate with no side effects in esophageal cancer treatment. It is also fascinating the hypothesis of using this bacterium and other probiotic *lactobacilli* for other cancer therapies.

## Figures and Tables

**Figure 1:** The effect of 5fu (a), *L. rhamnosus* supernatant (b), and whole-cell culture *L. rhamnosus* (c) on the cell viability of KYSE-30 cells.

**Figure 2:** Graph of the expression of Wnt signaling pathway genes. Each column indicates the fold change of expression value (2^−∆∆Ct^) of the genes in individual cell line KYSE-30.

**Figure 3:** Tumor growth curve. The average volume of cells xenograft into nude mice from 1-5 days (a), 5-10 days (b), and 10-15 days (c) posttreatment.

**Figure 4:** Histological changes of esophageal cancer cases with different stages. (a) Complete tumor necrosis magnification 10 (on the 5th day of sampling). (b) Undifferentiated tumor magnification 4 (on the 10th day of sampling). (c) Complete tumor necrosis magnification 40 (CFS and whole-cell culture of *L. rhamnosus*). (d) Overview tumor and necrosis magnification.

**Figure 5:** The effect of 5fu, *L. rhamnosus* supernatant, and *L. rhamnosus* whole-cell culture on nude mice tumor necrosis. Values are expressed as mean ± SEM. ^∗∗^*P* < 0.01.

**Table 1:** Primer sequences used for real-time PCR.

Seq name	Sequence
*β*-Actin, forward	GCCTCGCCTTTGCCGAT
*β*-Actin, reverse	TTCTGACCCATGCCCACCAT
APC, forward	AGACTGGTATTACGCTCAACTTC
APC, reverse	CTGGCTATTCTTCGCTGTGC
*β*-Catenin, forward	GGTGCTATCTGTCTGCTCTAGTAATAAG
*β*-Catenin, reverse	CCTTCCATCCCTTCCTGTTTAGTTG
GSK3B, forward	ACTTCACCACTCAAGAACTGTCAAG
GSK3B, reverse	TGTCCACGGTCTCCAGTATTAGC
LEF1, forward	GACAAGCACAAACCTCTCAG
LEF1, reverse	TTATTTGATGTTCTCGGGATGG
WNT1, forward	GGCTGGGTTTCTGCTACG
WNT1, reverse	TTCACAATACCCCACCATCG
Fzd1, forward	CTCCTACCTCAACTACCACTTC
Fzd1, reverse	CACTGACCAAATGCCAATCC
MYC, forward	AGCGACTCTGAGGAGGAACA
MYC, reverse	GACCAGTGGGCTGTGAGGA
Tcf7, forward	CGACCGCAACCTGAAGACA
Tcf7, reverse	AGTACTTGGCCTGCTCTTCTC
Cyclin D1, forward	CAAGTGTGACCCGGACTGC
Cyclin D1, reverse	CTCCTCTTCCTCCTCCTCGG
LRP5, forward	CGGCAGAAGGTGGTGGAG
LRP5, reverse	CAGCGAGTGTGGAAGAAAGG
LRP6, forward	GAACCTTCAAGAATACAGACAGCAC
LRP6, reverse	GCCAAGCCACAGGGATACAG

## Data Availability

All data are included in the manuscript.

## Abbreviations

CFS: Cell-free supernatant
ESCC: Esophageal squamous cell carcinoma
DMSO: Dimethyl sulfoxide
A&H: Hematoxylin-eosin
FBS: Fetal bovine serum
cDNA: Complimentary DNA.
